# Identification and Characterization of Cells with Cancer Stem Cell Properties in Human Primary Lung Cancer Cell Lines

This article has been retracted.

**DOI:** 10.1371/journal.pone.0057020

**Published:** 2013-03-04

**Authors:** Ping Wang, Quanli Gao, Zhenhe Suo, Else Munthe, Steinar Solberg, Liwei Ma, Mengyu Wang, Nomdo Anton Christiaan Westerdaal, Gunnar Kvalheim, Gustav Gaudernack

**Affiliations:** 1 Department of Immunology, Institute for Cancer Research, Oslo University Hospital, Radiumhospitalet, Oslo, Norway; 2 Department of Cellular Therapy, Oslo University Hospital, Radiumhospitalet, Oslo, Norway; 3 Cancer Stem Cell Innovation Centre, Oslo, Norway; 4 Department of Pathology, Oslo University Hospital, Radiumhospitalet, Oslo, Norway; 5 Department of Tumor Biology, Institute for Cancer Research, Oslo University Hospital, Radiumhospitalet, Oslo, Norway; 6 Department of Thoracic Surgery, Oslo University Hospital, Rikshospitalet, Oslo, Norway; 7 Department of Radiation Biology, Institute for Cancer Research, Oslo University Hospital, Radiumhospitalet, Oslo, Norway; 8 Faculty of Medicine, University of Oslo, Oslo, Norway; 9 Department of Hematology, Henan Tumor Hospital, Zhengzhou, People's Republic of China; The University of Texas M.D Anderson Cancer Center, United States of America

## Abstract

Lung cancer (LC) with its different subtypes is generally known as a therapy resistant cancer with the highest morbidity rate worldwide. Therapy resistance of a tumor is thought to be related to cancer stem cells (CSCs) within the tumors. There have been indications that the lung cancer is propagated and maintained by a small population of CSCs. To study this question we established a panel of 15 primary lung cancer cell lines (PLCCLs) from 20 fresh primary tumors using a robust serum-free culture system. We subsequently focused on identification of lung CSCs by studying these cell lines derived from 4 representative lung cancer subtypes such as small cell lung cancer (SCLC), large cell carcinoma (LCC), squamous cell carcinoma (SCC) and adenocarcinoma (AC). We identified a small population of cells strongly positive for CD44 (CD44^high^) and a main population which was either weakly positive or negative for CD44 (CD44^low/−^). Co-expression of CD90 further narrowed down the putative stem cell population in PLCCLs from SCLC and LCC as spheroid-forming cells were mainly found within the CD44^high^CD90^+^ sub-population. Moreover, these CD44^high^CD90^+^ cells revealed mesenchymal morphology, increased expression of mesenchymal markers *N-Cadherin* and *Vimentin*, increased mRNA levels of the embryonic stem cell related genes *Nanog* and *Oct4* and increased resistance to irradiation compared to other sub-populations studied, suggesting the CD44^high^CD90^+^ population a good candidate for the lung CSCs. Both CD44^high^CD90^+^ and CD44^high^CD90^−^ cells in the PLCCL derived from SCC formed spheroids, whereas the CD44^low/−^ cells were lacking this potential. These results indicate that CD44^high^CD90^+^ sub-population may represent CSCs in SCLC and LCC, whereas in SCC lung cancer subtype, CSC potentials were found within the CD44^high^ sub-population.

## Introduction

The “cancer stem cell” (CSC) theory implies a hierarchical organization within the tumor in which CSCs represents the apex of the hierarchy. Similar to normal stem cells, CSCs have the capacity to undergo self-renewal as well as asymmetric cell division. These key features enable CSCs to initiate and maintain tumors. In addition to the classical term, i.e. CSC, various terms have been used in the recent scientific literature to describe essential characteristics of CSCs such as self-renewal and tumor initiating/maintaining property. Among others are such terms as tumor initiating cell (TIC), cancer initiating cell (CIC) and tumor propagating cell (TPC). In this report we will use the CSC term to characterize cells that were able to initiate and sustain tumor formation in animals and long-term liquid culture.

Current studies in the field of cancer stem cell research have provided increasing evidence for the existence and identification of CSCs using several specific biomarkers, such as CD44, CD133 and CD90. These markers have been widely accepted for isolation of CSCs in human haematological malignancies [1], [2] as well as in solid tumors [3]–[11]. Furthermore, CSCs have been found to be more resistant to conventional chemotherapy and radiotherapy than the major population of more differentiated cancer cells, indicating that the CSCs may remain in residual tumors after treatment and contribute to cancer recurrence and spreading. Therefore, new treatments targeting CSCs may potentially prevent tumor recurrence and prolong survival of patients. The epithelial-mesenchymal transition (EMT) plays an important role in embryonic development [12]. It causes epithelial cells to lose their epithelial behavior, changing their morphology and cellular properties to resemble mesenchymal cells [13]. EMT has been suggested to contribute to the invasive and metastatic growth of many types of cancers [14]–[17]. Recent study showed that stem cell-like cells from epithelial cancers having a mesenchymal phenotype express markers associated with EMT [15].

Lung cancer is the leading cause of cancer-related mortality worldwide, and has a poor prognosis with 5-year survival rates of approximately 15%. According to the histological heterogeneity, lung carcinomas are categorized into four major subtypes: small cell lung cancer (SCLC), squamous cell carcinoma (SCC), large cell carcinoma (LCC) and adenocarcinoma (AC). In this study, following the “Cancer Stem Cell” hypothesis, we focused on the identification and characterization of CSCs in above mentioned subtypes of lung cancer.

The cell surface marker CD133 has previously been identified as a reliable marker for CSCs in some of lung cancer subtypes [18]. However, the reliability of this marker as a CSC marker for lung cancer has recently been disputed [19]. Therefore, we focused on another marker, i.e. CD44, which has been suggested to characterize CSCs in breast, prostate, head and neck, colorectal, pancreatic and gastric cancers [3], [4], [9]–[11], [20].

In this study, we took advantage of the primary lung cancer tissues removed during resection and focused on establishing of PLCCLs from freshly isolated tumors. We assumed that PLCCL may provide a more representative and appropriate source of cancer cells that can be used for identification of cells or cell populations with stem cell-like properties. We first successfully established a panel of the primary lung cancer cell lines from freshly obtained specimens of the major subtypes of lung cancer. Based on detailed phenotypic and functional analysis of representative cell lines from SCLC, LCC and SCC, we provide evidence indicating that CD44^high^ population may harbour CSCs in these cancer subtypes. In addition, co-expression of CD90 further narrowed down population of CSCs in SCLC and LCC. The picture for AC, however, remains less clear, and at the present we have no convincing evidence that either of the markers, i.e. CD44 and CD90, is characteristic for CSCs in this particular cancer subtype.

## Materials and Methods

### Collection of tumor specimens and establishment of primary lung cancer cell lines

This study was approved by the Regional Ethical Committee and the Institutional Review Board of Oslo University Hospital and performed according to the guidelines of the Helsinki Convention. Upon signed informed consent, human lung cancer tissues were obtained from 20 patients with primary lung cancer (age range 55–81 years) undergoing lobectomy or pneumonectomy at Oslo University Hospital from July 2007 to October 2009. Histological diagnosis was determined based on microscopic features of carcinoma cells (**Table 1**).

**Table 1:** Summary of the primary cultures included in this study.

Code No	Surgery date	Patient sex/age(years)^#^	PLCCL	Tumor type	Diagnosis pTMN
1	03.07.2007	M/70	LC003	AC	T1N0MXG2
2	18.07.2007	M/61	LC005	AC	T2N0MXG1
3*	25.07.2007	F/63	LC007	AC	T2N0MXG4
4	04.02.2008	M/73	LC013	AC	T3N1MXG3
5	06.02.2008	F/69	LC014	AC	T1N0MXG3
6	12.03.2008	F/72	LC016	AC	T2NxM1G2
7	29.09.2009	M/81	LC024	AC	T1N0MXG2
8	12.03 2008	M/80	LC017	SCC	T2NXMXG2
9	12.03.2008	M/71	LC018	SCC	T2N0MXG4
10	16.06.2008	M/56	LC019	SCC	T3N2MXG2
11*	21.07.2008	M/68	LC021	SCC	T2N2MXG2
12	23.07.2008	M/67	LC022	SCC	T2N0MXG2
13	21.08.2008	M55	LC023	SCC	T1N2MXG2
14*	24.07.2007	M/62	LC006	LCC	T2N1MXG4
15*	09.07.2007	F/71	LC004	SCLC	T1N0MXG2

# M, male; F, female.

* Primary cell lines highlighted in blue were used for further characterization.

Freshly obtained tumour tissue (within 1–2 hours after surgical removal) was washed in RPMI-1640 medium (Invitrogen, USA) containing penicillin-streptomycin (PS, penicillin 100 U/ml and streptomycin 100 μg/ml; Lonza, Belgium). Blood vessels and connective tissue were carefully removed and the cancerous part was then minced into small pieces less then 1 mm^3^ using scalpel, followed by extensive washing in RPMI-1640 medium and centrifugation at 300 g for 5 min. Finally, the cells were re-suspended in RPMI-1640 medium containing collagenase II (Invitrogen, USA) at the concentration of 200 U/ml and digested for 2–4 hours at 37°C in a humidified incubator. The enzymatic digestion was stopped when most of the cells were in the single cells suspension. Following washing in RPMI-1640 and 3x centrifugation at 300 g for 5 minutes, cells were transferred into standard tissue culture coated flasks (Corning Life Sciences, USA) and cultured in the Defined Keratinocyte-Serum Free Medium (DK-SFM) supplemented with L-glutamine (Invitrogen, USA), EGF 20 ng/ml, basic-FGF 10 ng/ml (PeproTech Inc., USA), 2% B27 (Invitrogen, USA), PS and amphotericin B (0.25 μg/ml; Invitrogen, USA). The cultures of all PLCCLs were maintained at 37°C in a humidified incubator with 5% CO_2_. Culture medium was changed every 2–3 days. Cells were passaged after detachment with TrypLE™Express (Invitrogen, USA), when the cells reached 80–90% confluence. All the studies were performed with the initial five passages of established PLCCLs.

### Isolation of nucleic acid and DNA fingerprinting assay

To establish a genetic fingerprint for each of the new cell lines, DNA fingerprinting assay was performed on the representative PLCCLs (LC004, LC006, LC007 and LC021) as well as on a re-established cell line from xenograft of LC021. Genomic DNA was isolated from Dulbecco's phosphate-buffered saline (DPBS, Invitrogen) washed cell pellets. Total genomic DNA was obtained using NucleoSpin Tissue kit (Macherey-Nagel, Germany) according to manufacturer's protocol. The identity of the DNA profiles was determined by STR profiling using Powerplex 16 System (Promega, Madison, WI). This kit amplifies 15 STR loci and amelogenin for gender identification: Penta E, D18S51, D21S11, TH01, D3S1358, FGA, TPOX, D8S1179, vWA, Amelogenin, Penta D, CSF1PO, D16S539, D7S820, D13S317 and D5S818. The PCR products were size determined in a MegaBace 1000 (Applied Biosystems, USA) using the software Fragment Profiler (GE Healthcare). These fingerprints were then compared to DNA profiles in a fingerprint database of previously established lung cancer cell lines to ensure their uniqueness.

### Immunohistochemistry

The primary cultured lung cancer cell lines were embedded into paraffin blocks by the following method: cells from the liquid culture were detached and washed with DPBS and subsequently centrifuged at 300 g for 5 minutes. The supernatant was carefully removed before 3 drops of plasma and 2 drops of thrombin were added and mixed by tube rotation. Buffered formalin (4%) was added after the mixture was coagulated. The coagulated mass was then placed in linen paper before being embedded in paraffin blocks by standard procedure. Some sections were stained with Hematoxylin and Eosin (H&E) to assess cellular morphology, while other sections were used for immunohistochemistry (IHC) analysis. Four micrometer thick sections were dewaxed and hydrated in graded ethanol. To unmask the epitopes, sections were then microwaved in different buffers optimised for different antibodies. Low pH 10 mM citrate buffer (pH  = 6.0) was used for antibodies P53, Ber-EP4 and CD44. To inhibit the endogenous peroxidase, the sections were incubated with 3% hydrogen peroxide (DakoCytomation, USA) for 5 minutes at room temperature (RT). Sections were then incubated with primary mouse anti-human P53, CD44 and Ber-EP4 (DAKO, 1∶1000, 1∶100 and 1∶300 dilutions, respectively) and CD133 (Miltenyi biotec, clone AC133/1 1∶40 dilution) antibodies for 30 minutes at RT followed by incubation with corresponding secondary antibodies for 30 minutes at RT and stained with 3,3′-diaminobenzidine tetrahydrochloride (Dako EnVision™+System Peroxidase (DAB) (K4007, DakoCytomation, USA)) before they were counterstained with hematoxylin, dehydrated and mounted in Diatex. All sections were rinsed thoroughly with TBS-Tween washing buffer (Dako Cytomation, USA) after each incubation step. Sections from paraffin blocks containing human seminoma and breast cancer specimen were used as positive controls for antibodies P53, Ber-EP4 and CD44, respectively; Sections from the paraffin block containing colon cancer cell line CaCo-2 were used as positive control for CD133 antibody. Isotype control antibodies at the same concentration were used as negative controls. All controls were performed and the antibody reactivity was verified before experimental applications of antibodies. Each stained section was reviewed independently by two pathologists.

### Animal experiments

All animal experiments were approved by and performed according to the guidelines set by the Animal Research Ethics Board at University of Oslo. Female NOD/SCID mice (NODSC-M-F/M-M Homozygous NOD/mrkBOMTac-Prkdcscid; Taconic, Denmark) were purchased. After being kept in quarantine one week for monitoring in the sterile environment of the animal facility in the Oslo University Hospital, Rikshospitalet, 4–5 weeks old NOD/SCID mice were used in all experiments. To assess the tumorigenicity of established PLCCLs, 3×10^6^ cells of each cell line suspended in DK-SFM were inoculated subcutaneously into the right flank of NOD/SCID mice (3 mice in each group) at a maximum volume of 100 µl. The mice were inspected twice a week and tumor size was measured with callipers. Mice were sacrificed by cervical dislocation when the size of the tumor reached a diameter of 15 mm. Xenografts were then removed and used for histological analysis and establishing of liquid cell cultures. Serial xeno-transplantations were performed with the LCC LC006 cell line by implanting pieces of the primary xenograft subcutaneously into secondary recipient NOD/SCID mice. Xenografts derived from each passage were taken out and fixed in 4% buffered formalin for histological analysis.

### Flow cytometry analysis and Fluorescence-Activated Cell Sorting (FACS)

Flow cytometry analysis was performed on PLCCLs at logarithmic growth phase. Cells were first detached with TrypLE™Express and washed with DPBS. Re-suspended cells were counted and transferred into 75 mm polystyrene round-bottom test tubes (BD Falcon, USA) at a cell concentration 1×10^6^ cells/ml, and subsequently stained with antibodies at dilutions determined by previous titration. Human immunoglobulin staining buffer (DPBS+0.1% human serum albumin (Octapharma, Stockholm, Sweden)) and 5 µL of 10 mg/ml gamma globulin (Gammagard, Baxter, UK) was added to the cells to block the FcR and minimize unspecific binding of antibodies. Fluorochrome coupled monoclonal antibodies (mAbs) were added to the test tubes at saturating concentrations and the cells were incubated for 20 minutes on ice avoiding light exposure. A screening for markers was performed with a panel of mAbs (see detailed data in Table 2) on four PLCCLs representing each lung cancer subtype. Cells stained with isotype-matched mAbs (BD Pharmingen, USA) served as negative controls. Different populations of cells were sorted based on the expressions of CD44 alone, or in combination with CD90 using a FACSAria II cell sorter (Becton Dickinson, Franklin Lakes, NJ). Flow data were acquired on the FACSAria II or LSR II cytometer (Becton Dickinson, Franklin Lakes, NJ). The results were analyzed using the BD FACSDiva software (Version 6.1.3). The viability of sorted cells was routinely checked using Trypan blue (Invitrogen, USA) staining and usually was >70%.

**Table 2:** Antibodies used in flow cytometry analysis.

Antigen	Conjugate	Clone	Source	Volume
CD15	APC	HI89	BD	20 µl
CD24	PE	ML5	BD	20 µl
CD29	PE	MAR4	BD	20 µl
CD31	PE	WM59	BD	20µl
CD34	PE, APC	563	BD	20 µl
CD44	FITC	G44-26 (C26)	BD	20 µl
CD45	FITC, PerCP	HI30,2D1	BD	20 µl
CD49b	PE	12F1	BD	20 µl
CD49f	PE-Cy5	GoH3	BD	20 µl
CD90	APC	5E10	BD	5 µl
CD142	PE	HTF-1	BD	20 µl
CD117	PE, PerCP-Cy5.5	YB5. B8,104D2	BD	5 µl, 20 µl
CD166	PE	3A6	BD	20 µl
CD184	PE	12G5	BD	20 µl
CD326	APC	EBA-1	BD	5 µl
CD133/1	APC	AC133	Miltenyi Biotec	10 µl
CD133/2	PE	293C3	Miltenyi Biotec	10 µl

FITC, fluorescein isothiocyanate; PE, phycoerythrin; PerCP, peridium chlorophyll protein; APC, allophycocyanin; Cy, cyanine dye.

### Cell proliferation assay

FACS sorted CD44^high^ and CD44^low/−^ cells at density of 150 or 500 cells per well were plated in triplicate in 200 µl DK-SFM with supplements in standard coated 96-well plates. Wells containing medium only were used as a background negative control. The cells were allowed to adhere at 37°C in a 5% CO_2_ humidified incubator for one day before they were used in the proliferation assay. Cell proliferation was measured during the following 8 days using CellTiter 96® AQueous One Solution Cell Proliferation Assay kit (Promega, Madison, WI) according to the protocol provided by the manufacturer. Absorbance at 490 nm was measured on a Wallac Victor2 plate reader (Perkin Elmer, Waltham, MA). The growth curves were drawn according to the mean value of absorbance, related to the background.

### 2 dimensional (2D) single cell colony forming and heterogeneity assay

CD44high and CD44^low/−^ cells from the SCLC cell line LC004 and the LCC cell line LC006 were sorted and seeded at a single cell per well into standard coated 96 well plates containing 200 μl DK-SFM supplemented with EGF 20 ng/ml, basic-FGF 10 ng/ml, and 2% B27. Single cell plating was validated by phase-contrast microscope (Nikon, Germany). Cultures were kept at 37°C in a 5% CO2 humidified incubator. After 2 weeks the number of positive wells containing colonies was counted and morphological characteristics of the colonies were evaluated. To study self-renewal and differentiation of single cells, the colonies of different types i.e. holoclones, meroclones and paraclones, were subjected to serial passages by picking and re-seeding them first into 24-well, then 6-well plates (Corning Life Science, USA), and eventually into the flasks (Corning Life Science, USA) where they were further expanded. Colony growth in 2D single cell colony forming assay and the long-term liquid cultures derived from these colonies were observed using phase-contrast microscope (Nikon, Germany).

### 2D colony formation efficiency assay

FACS sorted CD44^high^, CD44^low/−^ and CD44^high^CD90^+^ and CD44^high^CD90^−^ cells from the cell lines SCLC LC004 and LCC LC006 were seeded in triplicates at a density of 200 cells per well into standard coated 6 well plate (Corning Life Science, USA) containing 5 ml DK-SFM with supplements per well. The sorted cells were kept in culture at 37°C in 5% CO_2_ humidified incubator for ∼10 days. When the generated colonies were visible and contained >100 cells, the supernatant was aspirated and the wells were rinsed twice with DPBS, fixed in 4% buffered formalin for 15 min at RT followed by staining with crystal violet for another 15 min at RT. After rinsing away the dye, the colony number was counted and colony formation efficiency (CFE), i.e. the number of colonies per plated cell, was calculated and compared between different sub-populations.

### Spheroid formation assay

FACS sorted cells were seeded at density of 100 cells per well into ultra low attachment (ULA) 96 well plate (Corning Incorporated) containing 200 μl DK-SFM with supplements and cultured at 37°C in a 5% CO_2_ humidified incubator until cells started forming spheroids. The medium was changed every 2 days by carefully removing 50 μl of the upper layer of medium and replacing it with equal volume of fresh medium. The wells were inspected every 2 days using phase-contrast microscope. When the spheroids were big enough (most of the cell spheroids were >200 μm), they were counted and photographed (Nikon, Germany).

### RNA extraction and real-time PCR analysis

Total RNA was extracted from 10^5^ FACS sorted cells and subsequently reverse transcribed using Taqman Cell-to-CT kit (Applied Biosystems, USA) according to the protocol provided by the manufacturer. Real-time PCR was performed using Taq-Man Gene Expression Assay system (Applied Biosystems, USA) on 7900HT Fast Real-Time PCR System (Applied Biosystems, USA) according to the manufacturer's instructions and the data were analyzed by the SDS 2.3 Software (Applied Biosystems, USA). Each sample, including no template controls, was performed in duplicate. PCR reaction without template served as the negative control. Thermal cycling conditions were 50°C for 2 min and 95°C for 10 min followed by 40 cycles of 15 s at 95°C, followed by 1 min at 60°C. The expression levels were determined for the following genes *Nanog* (assay ID 8S02387400_gl), *Oct4* (assay ID Hs03005111_g1), *Sox2* (assay ID Hs01053049_sl), *E-Cadherin* (assay ID Hs01023895_m1), *N-Cadherin* (assay ID Hs00169953_m1), *Vimentin* (assay ID Hs00958111_ml), *high mobility group AT-hook 2 (HMGA2)* (assay ID HS00171569_ml) and *phosphoglycerate kinase 1* (*PGK1*) (assay ID Hs99999906_m1). The expression of target genes was related to the expression of *PGK1* and normalized to the unsorted control cells using the ddCT method.

### Radiation sensitivity assay

FACS sorted cells were seeded at a density of 500 cells per well in duplicates in standard coated 96 well plates (Corning Incorporated) containing 200 μl DK-SFM with supplements. After 24 hours of conventional incubation, cells in the monolayer cultures were irradiated at RT with doses of 1Gy, 2Gy and 4Gy, respectively using a Siemens Stabilipan X-ray unit, operated at 200 kV, 20 mA, with 0.5 mm copper filtration (Siemens, Germany). The cells were then cultured in regular culture conditions for 5 additional days with medium change every 2 days. The effect of irradiation on different cell populations was tested by the CellTiter 96® AQueous One Solution Cell Proliferation Assay as described above. The effect of irradiation on proliferation is given as the inhibition ratio and was calculated according to the formula: inhibition ratio  =  ((non-irradiated control well absorbance – irradiated well absorbance)/non-irradiated control well absorbance) ×100%.

## Results

### 1. Primary lung cancer cell lines

To provide a basis for the present study, a novel, robust method for culture of lung cancer cells from freshly resected lung carcinomas was established (see material and methods). Fifteen primary lung cancer cell lines were successfully established from 20 lung cancer tissues removed. These included 7 ACs, 6 SCCs, 1 LCC and 1 SCLC (**Table 1**). The success-rate of establishing primary cultures was 75%. The majority of failures occurred in the first part of the study, before optimal concentrations of the growth factors had been determined. The DK-SFM did support the selective growth of typical epithelial cells, clearly inhibiting the growth of co-existing fibroblasts. This was in contrast to cultures containing serum used in the beginning, where rapid overgrowth by fibroblasts occurred (data not shown). Monolayer cells with typical epithelial morphology were obtained at very high purity in each of the established PLCCLs (**Figure 1**). The primary cell lines maintained under these conditions were passaged for multiple generations with the longest passage so far over 30 generations, without any sign of growth decline.

**Figure 1:** Typical epithelial cells were obtained at high purity under the serum-free condition. **A.** The SCLC cell line LC004; **B.** The LCC cell line LC006; **C.** The AC cell line LC007; **D.** The SCC cell line LC021. All the representative images were from primary cultured lung cancer cell lines at the second passage. Photomicrograph magnification, ×200.

To ensure that the established cell lines were of unique origin and not contaminated by previously established cell lines [21], DNA profiles using a set of highly polymorphic microsatellite markers were generated from a subset of the cell lines representing the four different types of lung cancer. The results demonstrated that the four cell lines were unique and unrelated (Table Sl).

### 2. Phenotype of PLCCLs and parental cancer tissues have similar/are comparable for expression of P53, Ber-EP4 and CD44

We focused our work on four PLCCLs representing the four lung cancer subtypes: the SCLC cell line LC004, the LCC cell line LC006, the AC cell line LC007 and the SCC cell line LC021. From the selected representative PLCCLs, we prepared paraffin blocks, and sections from these cell lines were stained with H&E. Morphological evaluation of the PLCCLs confirmed their epithelial origin with signs of malignant transformation. Moreover, the primary cell lines derived from each of the four lung cancer subtypes were morphologically heterogeneous both at the cellular and nuclear level (**Figure 2A**).

**Figure 2:** Comparison of morphological and phenotypic features between the PLCCLs and corresponding tumor tissues. **A.** H&E staining of the 4 representative primary lung cancer cell lines for different lung cancer subtypes: the SCLC cell line LC004; the LCC cell line LC006; the AC cell line LC007 and the SCC cell line LC021. The cells derived from the four subtypes of lung cancer showed heterogeneity in cellular and nuclear morphology. Cells of each primary cell line had epithelial morphology. Photomicrograph magnification, ×200. **B.** Analysis the expression of P53, Ber-EP4 and CD44 in the 4 primary cell lines and their corresponding archival patients' tumor tissues. All the primary cell lines investigated showed diffuse positive staining for P53 except the original SCC tissue of cell line LC021. Epithelial membrane antigen Ber-EP4 was widely positive in all the original lung cancer tissues and diffuse positive in all the primary cell lines. CD44 showed diffuse positive staining with different intensity in the primary cell lines and their corresponding archival patients' cancer tissues except weakly positive in the original tumor tissue of the AC cell line LC007. Sections from paraffin blocks containing human seminoma and breast cancer specimen were used as positive controls for antibodies P53, Ber-EP4 and CD44, respectively. Photomicrograph magnification, ×200.

Tumor-suppressor protein P53 mutations is a hallmark of cancer and is generally up-regulated [22]. We next compared expression levels of P53 in serial sections from the archival patients' tumor tissues and the newly established PLCCLs using IHC. All four PLCCLs showed diffuse positive staining for P53. The same type of staining was observed in the original patient's cancer tissue with the exception of the SCC parental tissue, which was negative for P53 (Figure 2B). Interestingly, the cell line derived from the SCC (LC021) expressed P53. The expression levels of the Ber-EP4 and CD44 were investigated in the same way. The archival patients' tumor tissues and their corresponding PLCCLs showed broadly positive staining for the pan-epithelial marker Ber-EP4. Diffuse positive staining with different intensity in the archival patients' tumor tissues and their corresponding cell lines was seen with CD44 staining, except for the AC parental tumor tissue, which was weakly positive over most of the section studied (Figure 2B, Table S2). Expression of CD133 in the parental tumor tissues was also investigated by IHC staining. CD133 displayed a more variable pattern, with all the parental tumors being negative, except the SCLC (LC004) where expression in isolated areas was observed (data not shown). All PLCCLs derived from the corresponding parental cancer tissues were uniformly negative for CD133 expression by IHC staining.

Taken together the summarized experiments suggest that the PLCCLs in early passages (up to 5) are representative of the parental tumor tissue in all four cancer subtypes.

### 3. Primary cultures of lung cancer cells are as tumorigenic as xenotransplants

Malignant potential of the PLCCLs was investigated in an experimental animal model. A tumorigenesis assay was performed on 5 to 6-week old female NOD/SCID mice. Seven of the PLCCLs were tested in early passages and all were able to generate xenografts within 3 weeks after injection. The four cell lines SCLC LC004-P4, LCC LC006-P2, SCC LC021-P2 and AC LC007-P3, were chosen for further studies, propagating subcutaneous bulk tumors in 2/2, 3/3, 2/2 and 2/2 animals, respectively. Moreover, we were able to re-established PLCCLs *in vitro* from the xenografts taken from these animals (**Figure S1**). In addition, DNA fingerprinting was useful to track individual cell lines from the xenografts of LC021 (**Table S1** and **Figure S1**).

Based on these results we conclude the PLCCLs with the tumorigenesis capacity in immunodeficient mice can easily and reproducibly be generated from all four subtypes of lung cancer and propagated in *in vitro* liquid culture.

Secondary xeno-transplantation was performed by implanting subcutaneously pieces of the primary LCC xenograft (LC006) into secondary recipient. Primary recipient transplanted with LC006 cells revealed lung metastasis in addition to subcutaneous tumor. However, in the following serial xeno-transplantations, tumors were formed only subcutaneously. When morphological features of the PLCCL and the serial xenografts and parental tissues were compared, they displayed high similarity supporting the observation that PLCCLs and xenotransplants represent the original tumor.

### 4. Expression of CSC associated cell surface markers is dynamic in the long-term culture of PLCCLs

To identify subpopulations of putative lung cancer stem cells in the primary cancer cell lines, we investigated the expression of a broad panel of markers previously described as differentially expressed in a variety of human cancer stem cells. Data from six representative PLCCLs analyzed at different passages are given in **Table S3**. The expression profile revealed a variable pattern with some common features. In two cell lines (SCLC LC004 and SCC LC021) tested repeatedly the phenotype shifted during long term *in vitro* culture (Table S3). Some markers (CD29, CD49b and CD49f) were uniformly expressed at high levels in all passages and all cell lines studied, while others, such as CD44, CD166 and CD142, showed a higher expression in later compared to earlier passages. The opposite was observed for CD90 and CD326 expression, where the proportion of positive cells diminished with increasing passage number. Interestingly, distinct minor subpopulations expressing CD117, CD184 and CD15 were present in each of the cell lines tested. CD24 and CD326 showed variable expression level in different PLCCLs. The expression of CD133 was low, as tested by two different antibodies, and varied between 0–2.4% confirming the results obtained by IHC.

Thus, the expression level and the frequency of CD44 and/or CD90 positive sub-populations was dynamic, revealing differential expression of the antigens at different time points. These distinct changes that occurred during long-term culture indicate either possible selection of certain sub-populations in long-term culture or response to *in vitro* culture conditions.

All in all, our results clearly show that multiple cell surface antigens described to be differentially expressed in human CSCs, were also expressed on established PLCCLs, independent of the cancer subtype.

### 5. CD44^high^ cells from primary SCLC and LCC primary cell lines harbour cells with CSC characteristics

CD44 has been reported as a candidate CSC marker in many types of cancer [3], [4], [9]–[11]. All our PLCCLs expressed CD44 (Table S2). The flow cytometry analysis revealed the existence of distinct sub-populations with differential expression of CD44: a small sub-population of CD44high cells could be identified in both the SCLC cell line LC004 and the LCC cell line LC006, representing 6.63% (Figure 3A) or 2.79% of total cells (Figure 3B), respectively. Similar results were obtained for cell lines AC LC007 and SCC LC021 (Percentage of CD44high cells was 6.69% and 14.95%, respectively) (Figure 3C, D). The main cell population was either negative or weakly positive for CD44. To investigate possible functional differences between these subpopulations, CD44high and CD44low/− cells of SCLC LC004 and LCC LC006 were FACS-sorted and tested in several functional assays. The results from the colony formation efficiency assay suggest that CD44high cells from the SCLC LC004 and LCC LC006 cell lines have a significantly higher potential to form colonies compared to CD44low/− cells (data not shown and Figure 4A). The fact that CD44high cells formed bigger colonies suggests that CD44high cells from LC006 cell line proliferate more vigorously and for longer time than cells with low expression or negative for CD44.

**Figure 3:** Identification of CD44^high^ cells in the PLCCLs by flow cytometry analysis. A small sub-population of CD44^high^ cells could be identified in the SCLC cell line LC004 (6.63%) (**A**); the LCC cell line LC006 (2.79%) (**B**); the AC cell line LC007 (6.69%) (**C**) and the SCC cell line LC021 (14.95%) (**D**), respectively. Left panel: isotype control Ab; right panel: CD44 Ab. Data shown are from representative experiments (n>3).

**Figure 4:** Comparison of colony forming potential of different cell sub-populations from PLCCLs by colony formation efficiency assays. **A.** Comparison of FACS sorted CD44high and CD44low/− cells from the LCC cell line LC006. Cells were seeded at 200 cells per well and grown in standard 6 well plates for ∼10 days. Upper wells: CD44high cells. Lower wells: CD44low/− cells. **B.** Comparison of FACS sorted CD44highCD90+ and CD44highCD90− cells from the SCLC cell line LC004 (upper plate) and the LCC cell line LC006 (lower plate). Cells were seeded at 200 cells per well and grown in standard 6 well plates for ∼10 days. In each 6-well plate: upper wells: CD44highCD90+ cells; lower wells: CD44highCD90− cells. X denotes empty wells.

To investigate the proliferative potential of single cancer cells from PLCCLs, we next performed a single cell colony formation assay. Colony formation was observed 7∼10 days following plating. Only the CD44^high^ cells from the two cell lines SCLC LC004 and LCC LC006 were capable of forming a full range of colonies: holoclones, which consisted of tightly packed small cells, paraclones representing loosely packed colonies and meroclones with characteristics between holoclone and paraclone. CD44^low/−^ cells did not form holoclones, but were able to form a few meroclones and paraclones (**Figure S2 and Table S4**). To further study self-renewal and differentiation potential of cells isolated from the different colony types, the single cell derived colonies were picked, expanded and maintained in common cell culture flasks for long-term serial passages. Only the cells from holoclones, which were derived from the sorted CD44^high^ cells, had potential to maintain *in vitro* long-term cultures. When re-seeded into the colony assays, these cells formed all three types of colonies. Paraclones and meroclones both from CD44^high^ and CD44^low/−^ sorted cells stopped proliferating after one passage (data not shown).

These results demonstrate that CD44^high^ cells from SCLC and LCC cell lines contain cells with self-renewal and long-term growth potential. These stem cell-like properties were found only in CD44^high^ expressing cells.

We next compared the spheroid formation potential of CD44^high^ and CD44^low/−^ cells under serum-free conditions. Sorted cells were seeded at the concentration of 100 cells per well in ULA 96-well plate. Development of spheroids was evaluated 2 weeks after plating. Seven of ten wells with CD44^high^ cells from the SCLC cell line LC004 and 6/10 wells with CD44^high^ cells from the LCC cell line LC006 were identified with spheroid formation. Wells containing CD44^low/−^ cells from both cell lines did not reveal any formation of spheroids, and the cells eventually died (**Figure S3**).

Finally, growth curves of cell line LCC LC006 were determined by the CellTiter 96® AQueous One Solution Cell Proliferation Assay. At the highest cell concentration tested (500 cells/well) no significant difference in the proliferation of CD44^high^ and CD44^low/−^ cells was observed (**Figure S4**). However, when cells were seeded at a lower density (150 cells/well) CD44^high^ cells demonstrated higher proliferative potential compared to CD44^low/−^ cells (**Figure S4B**). Taken together, these results indicate that CD44^high^ population harbour cells with stem cell-like properties.

### 6. The CD44^high^CD90^+^ phenotype identifies sub-population of cells with stem cell-like properties in the SCLC and LCC

In order to narrow down the phenotype of the CSC population, the expression of additional putative stem cell markers were investigated. The initial analysis of PLCCLs by flow cytometry suggested that both CD44^high^ and CD44^low/−^ populations could be further sub-divided based on CD90 expression, namely CD44^high^CD90^+^, CD44^high^CD90^−^, CD44^low/−^CD90^+^, and CD44^low/−^CD90^−^ sub-populations (**Figure 5**). Since CD44^low/−^ population did not seem to contain cells with stem cell properties, CD44^low/−^CD90^+^, and CD44^low/−^CD90^−^ cells were sorted as one CD44^low/−^ population irrespective of CD90 expression. We then repeated the experiments described above, now testing 3 different sub-populations. In the 2D single cell colony forming and heterogeneity assay, only the CD44^high^CD90^+^ cells from the SCLC LC004 and LCC LC006 cell lines were able to form all three types of colonies (**Figure 4B**). Importantly, the cells derived from holoclones of sorted CD44^high^CD90^+^ cells maintained long-term *in vitro* growth and formed all three types of colonies when re-plated. CD44^high^CD90^−^ cells from the SCLC cell line LC004 gave rise to a single holoclone. This clone, however, did not sustain cell growth for more than one generation (**Table S5**). Repeatedly, CD44^low/−^ cells from SCLC and LCC cell lines, were able to form only a few meroclones and paraclones, which were not able to sustain a long-term growth in liquid culture and stop proliferating after one passage. These data indicate that CD44^high^ cells from SCLC and LCC cell lines that co-express CD90 have stem cell-like characteristics and sustain cell growth in liquid culture.

**Figure 5:** Flow cytometry analysis of CD44 and CD90 expression in the PLCCLs. Staining by anti-CD44 FITC and anti-CD90 APC. All the cell lines showed heterogeneous staining and could be divided into 4 sub-populations: CD44^high^CD90^+^, CD44^high^CD90^−^, CD44^low/−^CD90^+^ and CD44^low/−^CD90^−^. For the SCLC cell line LC004 (**A**), the frequency of CD44^high^CD90^+^ cell was 16.6%, and the CD44^high^CD90^−^ cells was 8.2%. For the LCC cells line LC006 (**B**), the frequency of CD44^high^CD90^+^ cells was 1.1%, the CD44^high^CD90^−^ cells was 2.5%. For the AC cell line LC007 (**C**), the frequency of CD44^high^CD90^+^ cells was 9.4%, and the CD44^high^CD90^−^ cells was 23.4%. For the SCC cell line LC021 (**D**), the frequency of CD44^high^CD90^+^ cells was 2.3%, the CD44^high^CD90^−^ cells was 1.1%.

Above mentioned cell populations were also tested in the spheroid forming assay. Cell spheroids were detected in 8/10 wells with sorted CD44^high^CD90^+^ cells from SCLC LC004 (**Figure S5A**) and in 8/10 from LCC LC006 (**Figure S5B**) cell line. In contrast, only 1/10 wells with CD44^high^CD90^−^ cells of both cell lines formed spheroids. As expected, no spheroids were formed in the wells with CD44^low/−^ cells irrespective of CD90 expression supporting the data from the 2D colony forming assay. These results clearly indicate that the spheroid forming cells are mainly harboured within the CD90^+^ subpopulation of the CD44^high^ cells.

We also tested the spheroid-forming capacity of the CD44^high^CD90^+^, CD44^high^CD90^−^and CD44^low/−^ cell populations in the SCC cell line LC021. Here 10/10 wells of CD44^high^CD90^+^ cells formed spheroids (**Figure S6A**), but contrary to the results of the SCLC cell line LC004 and LCC cell line LC006, 9/10 wells with CD44^high^CD90^−^ cells also formed spheroids (**Figure S6B**). No spheroids were formed in the wells with CD44^low/−^ cells (**Figure S6C**). Taken together, these results indicate that cells with stem cell-like characteristics are enriched in the CD44^high^ population also in the SCC cell line LC021. CD90, however, may not enrich further for the cells with stem cell-like properties.

A CD44^high^CD90^+^ population was also identified in the AC cell line LC007. However, neither CD44^high^CD90^+^, CD44^high^CD90^−^ nor CD44^low/−^ cells formed spheroids. Since this cell line did not form spheroids under the defined culture conditions, we cannot conclude whether either of the markers, i.e. CD44 and CD90, is a stem cells markers in the tested AC cell line.

### 7. The CD44^high^CD90^+^ sub-population exhibits stem cell and EMT associated gene expression profile in LC004 and LC021 primary cell lines

The observations that some sub-populations sorted based on expression of CD44 and CD90 had stem cell-like properties, prompted us to investigate whether the expression of stem cell related genes, such as *Nanog*, *Oct4* and *Sox2*, was different in these sub-populations of the cell lines LC004, LC006 and LC021. Detectable expression levels of these genes were found in all the sorted sub-populations. Interestingly, the expression of *Nanog*, *Oct4* and *Sox2* were higher in the CD44^high^ population compared to the CD44^low/−^ population in all the examined cell lines (**Figure 6**). Furthermore, the expression level of *Nanog* and *Oct4* genes was higher in the CD44^high^CD90^+^ population compared to the CD44^high^CD90^−^ population in the cell lines LC004 and LC006 (**Figure 6A, B**). However, no differences in gene expression levels except *Nanog* were observed between CD44^high^CD90^+^ and CD44^high^CD90^−^ populations in the LC021 cell line (**Figure 6C**).

**Figure 6:** Analysis of the expression of stem cell and EMT related genes in different sub-populations from the PLCCLs. Detectable expression levels of the genes were found in all sorted sub-populations from the cell lines LC004 (**A**), LC006 (**B**) and LC021 (**C**). PCR reaction without template served as a negative control. The relative expression of target genes was related to the expression of *PGK1* and normalized to the unsorted control cells. X axis shows the target genes, Y axis shows the relative expression level (RQ). The error bars reflect the variation within the triplicates, *P*<0.05. (B). The FACS sorted cell sub-populations derived from the cell line LC006 were cultured in the serum-free culture system for 1–2 weeks and revealed different cell morphology for different sorted sub-populations: (a) CD44highCD90+ cells; (b) CD44highCD90− cells; (c) CD44low/−CD90+ cells, and (d) CD44low/−CD90− cells. Photomicrograph magnification, ×200.

CSCs are proposed to play an important role in cancer invasion and metastasis seeding. Increasing evidence shows that epithelial-mesenchymal transition may impose stem cell characteristics on tumour cells, and accordingly, stem cell-like cells from carcinomas have a mesenchymal phenotype and express markers associated with EMT [15]. Culture of the different sorted cell populations derived from the LC006 cell line in our serum-free culture system shows that the sorted cell populations display different cell morphologies (Figure 6B). For example, the CD44highCD90+ and CD44highCD90− cells have a mesenchymal morphology, while the CD44low/−CD90+ and CD44low/−CD90− cells grow as cobblestones, a hallmark of epithelial cells. Therefore, we examined the expression profiles of EMT associated genes N-Cadherin, E-Cadherin, Vimentin, and HMGA2 in the sorted sub-populations from the cell lines LC004, LC006 and LC021. Interestingly, higher expression of the mesenchymal marker genes N-Cadherin, Vimentin and HMGA2, accompanied by a decreased expression for the epithelial marker gene E-Cadherin was found in the CD44high population compared to the CD44low/− population in all three cell lines (Figure 6A, B, C). The expression level of N-Cadherin and Vimentin were higher in the CD44highCD90+ population compared to the CD44highCD90− population from the cell lines LC004 and LC021 (Figure 6A, C), however, this was not the case for the same populations derived from the cell line LC006 (Figure 6B). The expression level of HMGA2 was higher in the CD44highCD90+ population compared to the CD44highCD90− population in the cell line LC004 (Figure 6A), no difference was observed between the subpopulations CD44highCD90+ and CD44highCD90− of the cell lines LC006 and LC021 (Figure 6B, C).

Altogether, our results of stem cell and EMT associated gene expression profile indicate a higher stem cell-like potential for the CD44^high^ population for all the examined cell lines. Co-expression of CD90 further enriched putative lung CSCs in the cell lines LC004 and LC006.

### 8. CD44^high^CD90^+^ cells from LCC primary cell line display the highest resistance to radiotherapy

The resistance to irradiation of CD44high and CD44^low/−^ cells from the LCC cell line LC006 was compared in an X-ray radiation resistance assay. Five days post irradiation with different doses, CellTiter 96® AQueous One Solution Cell Proliferation Assay was performed to compare the difference in cell proliferation of irradiated monolayer cultures from different cell sub-populations. The inhibition ratio of X-ray to the cells was calculated. The CD44high cells were more resistant to irradiation at each dose tested (**Figure 7A**). To investigate whether resistance to irradiation was associated with the CD44highCD90+ phenotype, the same assay was applied to determine the relative resistance to irradiation of the four cell populations derived from the same cell line. Among the four sub-populations, CD44highCD90+ cells displayed the highest resistance to irradiation at each dose tested (**Figure 7B**). This result further supports the notion that CD44highCD90+ population is enriched for putative lung CSCs.

**Figure 7:** Relative irradiation resistance of different sorted cell populations from the cell line LC006. A. The relative resistance to irradiation of the FACS sorted CD44high and CD44low/− cells derived from the LCC cell line LC006 was compared in an X-ray radiation resistance assay. The inhibition ratios were compared among the different cell populations after irradiating the monolayer cultures at 1, 2, 3 and 4Gy. The CD44high cells displayed the higher resistance to X-ray radiation at each dose tested. *P*<0.01. **B.** relative resistance to irradiation of the four different FACS sorted cell populations derived from the LCC cell line LC006 was compared in an X-ray radiation resistance assay. Four populations: CD44highCD90+, CD44highCD90−, CD44low/−CD90+ and CD44low/−CD90− cells were sorted into 96-well plates at 500 cells per well in 10 replicates. The inhibition ratios were compared among the four sub-populations after irradiation of the monolayer layer of the cultures at 1, 2 and 4Gy. The CD44highCD90+ cells displayed the highest resistance to irradiation at 2 and 4G. *P*<0.01.

### 9. The primary cell lines from long-term cultures changed their morphological features and the phenotype with time

In order to study the potential changes of established primary cell lines during long-term culture *in vitro*, we monitored the morphology and phenotype in the cell lines LC004 and LC021 at different passages. Although these primary lung cancer cell lines can successfully sustain long-term *in vitro* culture (the longest passage so far is over 30 generations of LC006) without growth decline, we observed certain changes in cell morphology. Cells from the first several passages demonstrated predominantly epithelial-like morphology, and then, the cells showed the change to mesenchymal features. Thereafter, shift towards more stressed epithelial-like morphology was observed following prolonged *in vitro* liquid culture.

We further employed flow cytometry to monitor phenotypic changes of the LC004 and LC021 cells at different passages, focusing on the CD44 and CD90 expression. In early passages (within passage 5), the cultured primary lung cancer cells maintained a sub-population of CD44^high^CD90^+^ cells. In later passages, the expression level of the CD44^high^ cells markedly increased while the expression level of CD90 decreased. The majority of the cells thus moved to the CD44^high^CD90^−^ region (**Figure S7 A, B**).

Concomitant with the changes in phenotype, cells from early passages demonstrated better colony forming potential compared to cells from later passages, corresponding to the decrease in the CD44^high^CD90+ subset from the prolonged culture (**Figure S7 A, B**).

The changes of morphology and phenotype during passaging of the cell lines may be caused by selection of certain sub-populations with distinct properties in an *in vitro* culture environment.

## Discussion

Tumor growth is hypothesized to depend on CSCs within a tumor, which shares the similar self-renewal function and capacity to generate differentiated cells with their normal stem cell counterparts. These cells can be identified by tumor stem cell associated antigens and other markers. Identification of reliable markers for CSC/TIC, which can be detected by robust tests such as flow cytometry using monoclonal antibodies, may open new opportunities for early diagnosis and staging, as well as the identification of novel targets leading to improvement of treatment for cancer in the clinic. By the use of different surface markers, CSCs/TICs have been identified in a variety of human cancers including acute myeloid leukemia, brain tumor, breast cancer, colon cancer, pancreatic cancer and prostate cancer [1]–[11].

In 2005, bronchioalveolar stem cells (BASCs) localized at the bronchioalveolar duct junction were identified as the tumor initiating cells for adenocarcinoma in a mouse model [23]. Recent attempts to identify lung CSCs in humans have suggested that CD133 [18] and also CD44 independently [24] could define a cell population with CSC characteristics. Later, several lines of evidence indicated that the ability of CD133 expression to discriminate lung CSCs may have been overestimated [19]. This is in line with our own observations showing that CD133 expression on lung cancer cell lines may be gained upon culture of sorted CD133 negative subpopulations and lost upon culture of CD133 positive subpopulation (Ping et al. unpublished). In the present study we accordingly focused on differential expression of CD44 in 4 representative primary cancer cell lines established from freshly resected tumors.

In order not to be restricted by the low number of cells available from surgical specimens and to be able to perform consecutive and repeated experiments on cancer cells derived from the same primary sample, we choose to study primary cell lines, which may also more accurately represent the situation in the patient compared to cell lines that have been established decades ago. In the present study, we successfully established a panel of novel cell lines from the primary cultures directly from different subtypes of freshly resected primary lung tumors. We used early passages of the generated cell lines to isolate phenotypically distinct sub-populations with stem cell features from these cell lines.

CD44 has been identified as a CSC marker for many cancer types, including breast cancer [4], prostate cancer [11], colorectal cancer [3] and lung cancer [24]. Flow cytometry and immunohistochemistry analyses showed that all the primary cultured lung cancer cell lines expressed CD44, but with marked differences in intensities and frequencies. A series of experiments aimed to evaluate whether lung CSCs could be enriched by the expression of CD44, demonstrated that CD44high cells always showed a stronger proliferative potential than CD44low/− cells, and only CD44high cells in the LC004 and LC006 cell lines were enriched in cells that could form holoclones, meroclones and paraclones reported to be associated with cancer stem cells [25]. The CD44high cells could form cell spheroids, whereas CD44low/− cells lacked this potential. Moreover, the CD44high sub-population showed a more mesenchymal morphology than the CD44low/− population. Together these results indicated that CD44high expression was associated with several stem cell characteristics in cell lines both from primary SCLC and LCC. These results confirm and extend the finding reported recently [24], which were mainly based on studies of established non-small cell lung cancer (NSCLC) cell lines. We did not investigate the potential co-expression of CD133 on the CD44high subpopulation. Such a co-expression might have solved the apparent controversy regarding the role of these two markers on lung cancer stem cells. The main reason for not doing so was the absence of CD133 expression in the surgical samples and the corresponding low or absent expression in the early passages of the cell lines derived from these samples.

CD90 is a marker expressed in mesenchymal stem cell [26] and liver cancer stem cell [27]. We found that it is also expressed in the primary lung cancer cell lines. By further co-staining with CD44 and CD90, all four representative primary cultured lung cancer cell lines could be divided into 4 heterogeneous sub-populations: CD44highCD90+, CD44low/−CD90+, CD44highCD90− and CD44low/−CD90− cell populations. In the SCLC cell line LC004 and the LCC cell line LC006, CD44highCD90+ cells had much stronger colony and spheroid forming potential. The self-renewal and differentiation analysis, demonstrated that only CD44highCD90+ cells were capable of forming holo-, mero- and paraclones. All the holoclones from CD44highCD90+ cells could be serially passaged and were capable of giving rise to all the same set of clones, while the only holoclone developed from CD44highCD90− cells was only able to sustain one generation. These results indicate that CD44highCD90+ cells may be able to undergo asymmetric divisions, giving rise to mature cells with a limited life span [28]. Fitting with the other findings, CD44highCD90+ cells in the LCC cell line LC006 also showed the highest level of resistance to irradiation. For the lung squamous cancer cell line LC021, CD44high expression alone may be a stem cell marker, since no further enrichment for colony formation or clonal growth was observed when CD90 was included. For the AC cell line LC007, only marginal differences in colony formation was observed in the four different sub-populations (data not shown). We are therefore unable to make any firm conclusion about the role of CD44 or CD90 as CSC marker in AC. Taken together, these result therefore indicate that CSCs in the four main subtypes may differ considerably in their phenotype.

Increasing evidence shows a direct link between the EMT and CSCs. Both EMT and CSC are implicated in the generation of invasive cells and formation of distant metastases. Furthermore, CSCs have been found to express EMT associated genes in addition to stemness associated genes [15]. Our observation that CD44high cells exhibited an increased expression of EMT associated genes indicates that CD44high cells may play a key role in progression of SCLC and LCC. Interestingly, CD44+CD90+ cells isolated from human hepatocellular carcinomas demonstrated a more aggressive phenotype than single positive, here CD90+/CD44− cells, forming more metastatic lung lesions in immunodeficient mice [27], indicating an important role of CD44 also in this type of cancer. The high mobility group A2 gene (HMGA2) is abundantly expressed in embryonic stem cells [29]. Aberrant re-expression of HMGA2 is correlated with tumor aggressiveness in a variety of human cancers [30], [31]. Furthermore, there is an increased expression of HMGA2 in cancer cells with stem cell characteristics, and the expression increase upon EMT [32]–[33]. In our study, the expression of HMGA2 was increased in the CD44high population compared to the CD44low/− population in three cell lines investigated, consistent with the increase of other EMT associated genes and stem cell related genes in this population.

In CSC research, established cancer cell lines are widely used to isolate and identify CSCs. Although it is relatively easy to use established cancer cell lines that have been grown for a long time *in vitro*, the CSCs identified in such cell lines may not truly reflect all biological features of primary CSC due to culture adaptation and genetic alterations taking place during long-term culture under hyperoxic culture conditions. The robust method for generating such primary cell lines from surgical specimens of lung cancer and identification of lung CSCs in these cell lines may provide a valuable and unique tool for further studies. With more reliable biomarkers available, these cell lines can also be used for screening of panels of different drugs targeting CSC related pathways.

## Supporting Information

Figure S1 **The flow cytometry analysis of xeno-cell line LC021.** Xeno-cell line LC021 displayed a hierarchical organization similar to that found in primary cultures, CD44^high^CD90^+^ cells were found in xeno-cell line LC021. Anti-Tra-1-85 Ab was used to gate human cells; Anti-H2Kd Ab was used to gate mouse cells.
(TIF)

Figure S2 **Clonal heterogeneity assay of sorted cell populations from the cell lines LC004 and LC006.** Sorted cells were cultured under serum-free condition for 2 weeks after seeding of 1 single cell per well in 96-well standard plate. Two weeks later, heterogeneous colonies of distinct morphologies were identified in CD44high cell populations from the SCLC cell line LC004 (**A**) and the LCC cell line LC006 (**B**). **Left column:** Typical holoclones which are generally more round and tightly packed composed of homogenous cells. **Middle column:** meroclones which are colonies made of cells of intermediate morphology and cell numbers. **Right column:** paraclones which are irregular in shape and contain fewer and more elongated or flattened cells. Representative colony images were acquired at 100×.
(TIF)

Figure S3 **Potential of sorted CD44^high^ and CD44^low/−^ cells to form spheroids under serum-free culture condition.** Cells were seeded at 100 cells per well in ULA 96-well under serum-free condition. CD44^high^ cells of the SCLC cell line LC004 (**A**) and the LCC cell line LC006 (**C**) developed cell spheroids 7–10 days after plating, while CD44^low/−^ cells from both cell line LC004 (**B**) and LC006 (**D**) formed no spheroids. The assay was repeated twice with similar results. The photomicrograph shows representative sections of the wells. Photomicrograph magnification 200×.
(TIF)

Figure S4 **Proliferation of CD44high and CD44^low/−^ cells from the PLCCL LC006 at different cell concentrations and different time points. A.** Proliferation of sorted CD44high (blue line) and CD44^low/−^ (purple line) cells seeded at 500 cells per well in 96 well plate. **B.** Proliferation of sorted CD44high and CD44^low/−^ cell populations seeded at 150 cells per well under identical culture conditions. Data represent the mean value of at least three wells.
(TIF)

Figure S5 **Potential of sorted sub-populations from LC004 and LC006 PLCCLs to form spheroids under serum-free culture condition.** Four populations were sorted based on expression of CD44 and CD90 surface markers. Results are shown only for the CD44^high^CD90^+^ sub-population that had the potential to form spheroids. Sorted cells were seeded at 100 cells per well in ULA 96-well under serum-free condition. Cell spheroids were formed only in wells with CD44^high^CD90^+^ cells from LC004 (**A**) and from LC006 (**B**). Photomicrograph magnification 200×.
(TIF)

Figure S6 **Comparison of cell spheroid formation of different sub-populations from the LC021 under serum-free condition.** CD44^high^CD90^+^, CD44^high^CD90^−^ and CD44^low/−^ cell populations were sorted from the SCC cell line LC021. Spheroids were formed by CD44^high^CD90^+^ cells (**A**) and by CD44^high^CD90^−^ cells (**B**). None of spheroids was formed by CD44^low/−^ cells (**C**). Photomicrograph magnification 200×.
(TIF)

Figure S7 **Morphological and phenotypic changes of PLCCLs LC004 and LC021 upon long-term** ***in vitro*** **culture. A.** Monitoring of the morphology and phenotype of the cell line LC004 at different passages upon long-term *in vitro* culture. **a.** In early passages, the cultured cells predominantly demonstrated mesenchymal morphology, while a shift towards a more stressed epithelial-like morphology was observed following prolonged *in vitro* culture in serum free medium. Photomicrograph magnification 200×. **b.** Monitoring of the phenotypical changes of the LC004 cells at different passages, based on the expression level of CD44 and CD90 by flow cytometry. **c.** The charts showing the changes of phenotype (upper left and right), colony forming efficiency (lower left) and propagation (lower right) of the LC004 cells upon long term *in vitro* culture. **B.** Monitoring of the morphology and phenotype of the cell line LC021 at different passages upon long-term culture *in vitro*. **a.** Monitoring of the phenotypical changes of the LC004 and LC021 cells at different passages based on expression of CD44 and CD90 by flow cytometry. **b.** The charts show the changes of phenotype (upper left and right), colony forming efficiency (lower left) and propergation (lower right) of the LC021 cells upon long term *in vitro* culture.
(TIF)

Table S1 **DNA fingerprinting data on PLCCLs.**
(DOC)

Table S2 **Summary of immunoshistochemical analysis of P53, Ber-EP4, and CD44 of PLCCLs and their corresponding parental tumor tissue.**
(DOC)

Table S3 **Expression of a broad panel of cancer stem cell associated markers analyzed in six representative cell lines at different passages.**
(DOC)

Table S4 **Single cell 2D colony forming and heterogeneity assay.**
(DOC)

Table S5 **Single cell 2D colony forming and heterogeneity assay.**
(DOC)
